RETRACTED

# Affective Antidepressant, Cytotoxic Activities, and Characterization of Phyto-Assisted Zinc Oxide Nanoparticles Synthesized Using *Sanvitalia procumbens* Aqueous Extract

**DOI:** 10.1155/2022/1621372

**Published:** 2022-06-16

**Authors:** Yasir Rashid, Fozia, Ijaz Ahmad, Nisar Ahmad, Madeeha Aslam, Amal Alotaibi

**Affiliations:** ^1^Department of Chemistry, Kohat University of Science & Technology (KUST), Kohat, Pakistan; ^2^Biochemistry Department, Khyber Medical University Institute of Medical Sciences, Kohat, Pakistan; ^3^Basic Science Department, College of Medicine, Princess Nourah Bint Abdulrahman University, Riyadh, Saudi Arabia

## Abstract

Green synthesis of nanoparticles has emerged as an effective and environmentally friendly method. Therefore, the current investigation is based on the green synthesis of zinc oxide nanoparticles (ZnO-NPs) using plant extract of *Sanvitalia procumbens* (*S. procumbens*) that act as a capping and reducing agent. *S. procumbens* is a fast-growing shrub and densely available plant and may have potential to synthesize ZnO-NPs. The synthesized ZnO-NPs were characterized by different techniques, including Fourier transform infrared spectroscopy (FT-IR), UV-visible (UV-Vis), energy-dispersive X-ray (EDX), X-ray diffraction (XRD), and scanning electron microscopy (SEM). The UV-Vis spectrum at 350 nm revealed an absorption peak for the synthesis of ZnO-NPs. In addition, photoactive biomolecules of the prepared ZnO-NPs were identified by using FT-IR spectroscopy. Furthermore, the spherical geometry of ZnO-NPs was evaluated by SEM images. The synthesized ZnO-NPs were also used to enhance the antidepressant activity and exhibited a remarkable reduction in the time of immobility in tail suspension tests (TST) and forced swim tests (FST), as well as increased the BDNF levels in the brain and plasma. ZnO-NPs have a low risk of biocompatibility (cell visibility) at a concentration of 7 g/mL or below. The nanoparticles were biologically compatible when the concentrations were increased up to 11 *μ*g/mL. It was concluded that ZnO-NPs were investigated as a possible carrier for antidepressant drug delivery into the brain, and their excellent cytotoxic activity was evaluated by using the MTT assay to determine their biocompatibility.

## 1. Introduction

Nanotechnology is an innovative field of science that might have profound applications in different fields, such as energy, environment, and electronics. Nanoparticles established new properties at the nanoscale, including thermal conductivity, crystal structure, surface morphology, large surface area, charge, shape, and zeta potential, which allow them to be used in biotechnological and biomedical applications. Because of their unique properties, metal oxide nanoparticles are becoming incredibly common [1, 2]. Among various metal oxide nanoparticles, ZnO-NPs are the most notable metal oxide nanoparticles owing to their distinctive physical and chemical characteristics, with 60 meV and 3.3 eV of high exciton binding energy and direct band gap energy at room temperature, respectively. The ZnO-NPs have additional advantages over other oxide nanoparticles with regard to their existence of different sizes and shapes at room temperature and in the reverence for counterparts in terms of cost, lack of colouration, UV protection, and easy production procedure. Therefore, the multifunctional ZnO-NPs have been used in cosmetics, biomedicines, drug delivery systems, agriculture, and biosensors [3, 4]. In addition to these applications, recent studies have demonstrated that ZnO-NPs have a wide range of antibacterial effects on microorganisms which depend upon the size and the presence of visible light [5]. Furthermore, ZnO-NPs may also release reactive oxygen-containing species (ROSs) that contribute to their biomedical properties [6]. According to the US Food and Drug Administration (FDA), ZnO is considered a safe drug carrier system when the particles are larger than 100 nm, due to its biocompatibility [7, 8]. The cytotoxicity of ZnO-NPs for human healthcare systems is still being questioned, as nanoparticles possess different mechanisms of toxicity, including cell internalization, reactive oxygen species (ROS) production, and metal ion release that may have a different impact on human cells than the bulk material [9]. Previous investigation has revealed that the cytotoxicity of ZnO-NPs is not only dose-dependent but also exposed to size, morphology, and surface properties. Therefore, ZnO is used for targeted drug delivery, but it still has a cytotoxicity problem. Currently, ZnO-NPs have been used to solve this problem [10, 11]. Various methods are now available for the synthesis of ZnO-NPs, such as chemical, hydrothermal, precipitation, microwave, sonication, and solvothermal. These methods entail the use of extreme reaction conditions and hazardous chemicals resulting in environmental contamination and chemical toxicity. However, the need for environment-friendly protocols for the synthesis of nanoparticles developed interest in green synthesis approaches compared to traditional methods [12]. Thus, the synthesis of ZnO-NPs using plant extracts enhanced the biocompatibility of nanoparticles and also play an important role in different biomedical applications. The presence of various phytochemicals and enzymes (like organic acids, flavones, and quinones) in plant extract aids the reduction or oxidation of the precursor molecule to ZnO-NPs [13]. Recently, different groups have reported on the green synthesis of ZnO-NPs using plant extracts, including *Momordica charantia* [14] and *Azadirachta indica* (L.) [15] which act as a reducing and stabilizing agent.

RETRACTED

According to the World Health Organization, depression has become a life-debilitating psychiatric disorder that causes morbidity and mortality and affects over 200 million people worldwide [16]. The above disorder probably starts at a young age and has a negative impact on ability functions of peoples and is frequently chronic. As a result of these issues, depression is recognized as the major problem of disability in terms of the overall age lost due to the worldwide disability. The demand of therapeutic interventions for depression and other mental illnesses is increasing all over the world. It is really attributed to the decrease of the quality life and social interaction, as well as enhanced thoughts of suicide, that has significant risk of morbidity and mortality as well as cardiovascular disease. Depression is a severe brain disorder that adversely effects psychological, behavioral, and physical health and has significant economic and social consequences [17]. Several medicines are used to treat depression, including serotonin, tricyclic antidepressants, reuptake inhibitors, noradrenaline, and monoamine oxidase inhibitors. Besides these, they might have numerous detrimental effects like dry mouth, sleepiness, and stomach pain [18]. Therefore, medicinal-mediated nanoparticles may be used for the therapy of antidepressants that can significantly strengthen the health status of people suffering from depressive disorders. So, the current study was conducted for the synthesis of ZnO-NPs employing an aqueous extract of the plant and to assess their biomedical prospective in terms of their antidepressant activity.

According to the reported literature, it was confirmed that ZnO-NPs were not synthesized from the aqueous plant extract of *Sanvitalia procumbens* that act as a reducing and capping agent. The plant *S. procumbens* belongs to the Asteraceae family, which is one of the most essential plant families for ornamental, medicinal, dietary, and other aromatic purposes. Several studies highlighted the effectiveness of alkamide and terpenoid functional groups that are derived from medicinal plants used to cure stomach pain, indigestion, vomiting, diarrhea, dysentery, and other gastrointestinal disorders. Furthermore, it contains many beneficial phytochemicals such as terpenoids, phenolics, alkamides, and proteins [19–22] that might serve as stabilizing and reducing agents during ZnO-NP synthesis. Furthermore, the elemental composition, geometry, morphology, and optical study of synthesized AgNPs were carried out by using various techniques such as energy-dispersive X-ray (EDX) analysis, X-ray diffractometer, scanning electron microscope (SEM), Fourier transform infrared spectroscopy (FT-IR), and UV-visible spectrophotometry. The current research contributes to a superior comprehension of the molecular level green synthesis of ZnO-NPs that is necessary for the development and implementation of a large-scale production of nanoparticles. Moreover, the present study was used for the first time to assess their biological application via green-synthesized ZnO-NPs for antidepressant and cytotoxic activities using the MTT assay which was used to explore their implementation in the field of biomedicine.

RETRACTED

## 2. Material and Methods

### 2.1. Chemicals

The chemical ZnCl_2_·2H_2_O (Sigma-Aldrich) has a percent purity of 98%. The glucose and glutamine were used for the preparation of Dulbecco media. Streptomycin, penicillin, the drug fluoxetine hydrochloride (Sigma-Aldrich), dimethyl sulfoxide (DMSO), and 3-(4,5-dimethylthiazol-2-yl)-2,5 diphenyltetrazolium bromide (MTT) were used in the assay.

### 2.2. Plant Collection

The whole plant of *Sanvitalia procumbens* was accumulated in the month of December 2019, when plants were at a flowering or mature stage, from the region of Kohat, KPK, Pakistan. The plant was recognized by Dr. Nisar Ahmed, Department of Plant and Environmental Sciences, Kohat University of Science and Technology.

### 2.3. Plant Extraction

The plant was rinsed with distilled water to remove dust and debris and shade-dried at room temperature. Using a mortar and pestle, the dry plant was ground into fine powder. 10 g of the powder plant was poured into a conical flask containing 100 mL distilled water and agitated at room temperature for 72 hours on a rotatory orbital shaker. The mixture was then filtered with filter paper, and the filtrate was used for reduction of zinc ions.

### 2.4. Green Synthesis of ZnO-NPs

The ZnO-NP synthesis was achieved via the green synthesis procedure. 9 mL of aqueous plant extract was added to a 1 mL solution of ZnCl_2_·2H_2_O (0.5 M) in a dropwise manner and was constantly stirred at ambient temperature. The colour change was observed after 2 hours of the reaction mixture. The synthesized ZnO-NPs were subjected to centrifugation for 20 minutes at 6000 rpm. The ZnO-NPs were rinsed with distilled water and methanol to remove any trace of unbound phytoconstituents for 2-3 times. The powder form of ZnO-NPs was dehydrated in a clean oven at 50°C and was used for further analysis [23].

RETRACTED

### 2.5. Characterization of ZnO-NPs

Different techniques were used to characterize the synthesized ZnO-NPs, including UV-Vis, FT-IR, EDX, SEM, and XRD.

#### 2.5.1. Ultraviolet-Visible (UV-Vis) Spectroscopy

The reaction mixture of ZnO-NPs was used to analyze the formation of nanoparticles. UV-Vis spectroscopy was used to monitor the green-synthesized ZnO-NPs in a colloid solution that demonstrates the sharp peak of absorption because of the surface plasmon resonance (SPR) excitation. The colour of the aqueous extract plant/ZnCl_2_·2H_2_O mixture was changed and then checked by spectrophotometric (Shimadzu-UV-1800) analysis at wavelengths of 200–800 nm.

#### 2.5.2. Fourier Transform Infrared (FT-IR) Spectroscopy

The FT-IR (Bruker-Tensor 37) analysis was used for the identification of functional groups present in green-synthesized ZnO-NPs. Potassium bromide (KBr) was added to around 0.2 g of ZnO-NP powder and then deposited onto a disc at high pressure. The spectra of FT-IR were examined at a wavelength of 400-4000 cm^−1^ with a resolution of 4.0 cm^−1^.

#### 2.5.3. Scanning Electron Microscopy (SEM)

The shape and size of ZnO-NPs was investigated by employing SEM JSM5910 (JEOL, Japan). The image was obtained with a scanning electron microscope after using fine powder of ZnO-NPs at a 20 kV accelerating voltage.

#### 2.5.4. Energy-Dispersive Spectroscopy (EDX)

An energy-dispersive spectroscope (EDX) was used to detect the elemental compositions and surface shape of the synthesized ZnO-NPs, at 20 keV accelerating voltage.

#### 2.5.5. X-Ray Diffraction (XRD) Patterns

The X-ray diffraction pattern (XPERT-PRO) revealed the crystalline nature of ZnO-NPs synthesized by plant extract of *S. procumbens*. CuK*α* radiation was employed to detect the X-ray diffraction over the 2*θ* angle ranges from 10° to 90°. Both current and voltage were set at around 30 mA and 40 kV, respectively. The average size of nanoparticles was obtained by employing Equation (1), the Debye-Scherrer equation, as shown below:

(1) $$\begin{array}{c} D=\frac{0.9\lambda }{\beta \cos\theta }, \end{array}$$

where *D* denotes the average size of nanoparticle, 0.9 represents Scherrer's constant, *λ* corresponds to the X-ray wavelength used as 1.540 Å, *β* is FWHM (full width half maximum), and *θ* corresponds to Bragg's angle.

### 2.6. In Vivo Antidepressant Activity of ZnO-NPs

#### 2.6.1. Animals

The antidepressant activity of ZnO-NPs was examined in male Sprague Dawley rats (200 ± 20 g) which were easily accumulated from the National Institute of Health (Islamabad, Pakistan). Animals received adequate water and food to adapt to the environment of a laboratory under standard conditions, having a relative humidity of 40–60% and maintaining their temperature at 25 ± 0.5°C. The Ethics Committee of the Riphah Institute of Pharmaceutical Sciences and Institutional Research approved all experimental studies on animals in accordance with the Animal Welfare Act and NIH policy.

RETRACTED

#### 2.6.2. Experiment Design

The activity of the antidepressant was examined by using synthesized ZnO-NPs. For this experiment, rats were classified into five groups; 1^st^ group (control) consists of healthy rats that received saline, 2^nd^ group (depressive) consists of depressant rats that received saline, 3^rd^ group (depressive+ZnCl_2Chem_) consists of depressant rats that received 10 mg/mL ZnCl_2Chem_ dissolved in saline, 4th group (depressive+extract) consists of depressant rats that received 150 mg/mL plant extract in saline, and 5th group (depressive+ZnO-NPs) consists of depressant rats that received ZnO-NPs dissolved in saline 8 mg/mL on alternate days for a period of 14 days. The animals were exposed to behavioral and pretest analyses for 15 and 16 days, respectively. After that, a cardiac puncture was used to obtain blood from the animals, which was then centrifuged for 15 minutes at 3000 rpm to separate plasma. Each rat was sacrificed after blood was collected, and the brain was separated via decapitation and cleaned with normal saline. Finally, the concentration of BDNF in the supernatant plasma and brain was ascertained by utilizing an appropriate rat ELISA kit that was obtained from Elabscience Biotechnology Co., Ltd. (Wuhan, Hubei, China). Elabscience Biotechnology Co., Ltd. (Elabscience) is a high-biotech company that specializes in reagents for immunodiagnostic technology. It offers more than 20,000 products, including ELISA kits, antibody, and proteins [24]. The drug fluoxetine hydrochloride (Sigma-Aldrich) was used as reference standards for antidepressant activity.

#### 2.6.3. Behavioral Analysis

The tail suspension tests (TST) and forced swim tests (FST) were used to study the behavioral analysis of rats. An FST was conducted in a glass cylinder (21 × 21 × 50 cm) loaded up to 35 cm of water and kept at a temperature of 24 ± 1°C [25]. A pretest was performed by placing each rat in the cylinder for 15 minutes and then allowed to dry at room temperature. On an aforementioned day, each rat was placed in the cylinder for 5 minutes, and the time of immobility was recorded under the same conditions. The absence of movement to escape and float in water, as well as efforts like keeping their heads above the water level, was a prediction of immobility. After each swim, the water was changed to prevent behavioral changes caused by contamination. The TST experiment was carried out by suspending the tails of rats 50 cm above the ground using adhesive tape [26]. A climb stopper was placed around the tail to prevent rats from grabbing onto their tails. Time of immobility was investigated by the absence of escape behavior that was measured for each rat over a period of 6 minutes.

RETRACTED

#### 2.6.4. Quantification of BDNF Concentrations in Plasma and Brain Samples

The BDNF concentration (brain-derived neurotrophic factor) in brain and plasma samples attained from the animals after behavioral studies was determined via an ELISA kit (Elabscience Biotechnology Co., Ltd., Wuhan, Hubei, China). In order to accomplish this, cortices were removed from the brain samples, coagulated with PBS, and centrifuged for 15 minutes at 3000 rpm, and the filtrate was accumulated. According to the manufacturer's instructions, the BDNF concentration in the filtrate of the brain and plasma was finally ascertained through employing its respective rat ELISA kit (Elabscience Biotechnology Co., Ltd., Wuhan, Hubei, China).

### 2.7. Cytotoxic Activity of ZnO-NPs

#### 2.7.1. Cell Culture

The neuroblastoma (Neuro2A) cells were incubated in the modified Dulbecco's media (1 g/L glucose, 2 mM glutamine) with 10% FBS, 100 *μ*g/mL of streptomycin, and 100 *μ*g/mL of penicillin, at a temperature of 37°C and the atmosphere of CO_2_ with 5% moisture.

#### 2.7.2. Cytotoxic Evaluation

The cytotoxic evaluation of synthesized ZnO-NPs was analyzed by employing 3-(4,5-dimethylthiazol-2-yl)-2,5 diphenyltetrazolium bromide (MTT) assay. In simple words, cell suspension containing (200 *μ*L) was subjected to a 96-well tissue culture plate (1 to 104 cells/well) and heated at 37°C for 24 hours. After that, 50 *μ*L (0–600 *μ*g/mL) of the synthesized ZnO nanoparticles was applied in each well, and the plate was placed for 24 hours of incubation. In this, the identification of the cell suspension that was held in the culture medium was used as the control. The plate was then incubated for 4 hours at 37°C with 20 *μ*L of MTT-containing PBS buffer (5 mg/mL) added to each well. The optical absorbance of each well was measured at 542 nm using a microplate reader after 100 *μ*L of DMSO was added at the end of each well. The cell viability relative to the control group was expressed as a percentage [11].

## 3. Results and Discussion

### 3.1. UV-Visible Analysis of ZnO-NPs

Visual observation is the first indication for the formation of ZnO-NPs that is accompanied by UV-Vis analysis at different wavelengths ranging 200-800 nm to identify surface plasmon resonance (SPR). For the synthesis of ZnO-NPs, the transition of an electron from the valence band to the conduction band induced the characteristic peak. The plant-mediated green synthesis of ZnO-NPs was observed in UV-Vis spectra, which is shown in Figure 1. A significant absorbance peak at 350 nm, without any other peaks, confirmed that the existence of active biomolecules present in the plant extract helps in reduction and stabilization of ZnO-NPs. The following Equation (2) was used to calculate the band gap energy (*E*) for ZnO-NPs with a wavelength (*λ*) of 350 nm.

(2) $$\begin{array}{c} E=\frac{hc}{\lambda }, \end{array}$$

where *h* represents Planck's constant (6.626 × 10^−34^ kg m^2^/s) and the light velocity (3 × 10^8^ m/s) is denoted by *c*. The 3.54 eV was determined by calculating as the band gap energy for the NPs. The band gap of ZnO-NPs is characterized by performing UV-visible spectroscopy. Because of the smaller band gap, the electron is easily excited from the valence band to the conduction band. In the previous literature, it was also reported that by performing UV spectroscopy on ZnO-NPs, the band gap obtained was 3.29 eV. The band gap depends on various factors, including the grain size, oxygen deficiency, surface roughness, and lattice strain. These results are consistent with those of our previously reported green-synthesized ZnO-NPs via the *Rhazya stricta* plant extract, which showed SPR at 353 nm [4, 27].

RETRACTED

### 3.2. FT-IR Analysis of ZnO-NPs

The characterization of FT-IR was used to achieve the chemical structures as well as functional groups present in the *S. procumbens* plant extract and ZnO-NPs within the range of 500-4000 cm^−1^. The FT-IR analysis of the *S. procumbence* plant extract exhibits different bands in the regions of 3261, 1590, 1405, and 1033 cm^−1^ (Figure 2) that is comparable to those of our previously reported article [28]. The O-H stretching of carboxylic acid was related to the broad band absorption at 3261 cm^−1^, whereas the band at 1590 cm^−1^ corresponding to the stretching vibration of N-H is present in amines of proteins [29]. The C-N stretching vibration of amino acids is associated with the sharp intensity peak at 1405 cm^−1^, while the sharp peak at 1033 cm^−1^ can be correlated with the stretching vibration of C-O present in carboxylic acid, alcohols, and esters. The reduction in bands at 3216, 1560, 1397, 1024, and 871 cm^−1^ is due to the presence of phytochemicals present in the plant extract which help in the reduction of ZnO ions [30]. Therefore, we hypothesized that the biomolecules capped the ZnO-NPs and are also responsible for the formation of ZnO-NPs. The absorption band at 690 cm^−1^ indicates the successful synthesis that was confirmed by the ZnO bond. The FT-IR analysis showed that organic substances found in the *S. procumbens* plant extract play a significant role in the stabilization and reduction of green-synthesized ZnO-NPs.

RETRACTED

### 3.3. XRD Pattern of ZnO-NPs

The X-ray crystallography technique was used to evaluate the crystalline nature of ZnO-NPs within the range of 10-80 degrees at 2*θ*.  Figure 3 shows the XRD patterns of the sample that confirmed the crystal structure of ZnO-NPs having characteristic peaks 31°, 34°, 36°, 47°, 56°, 63°, and 67° at the 2*θ* position, correlated to the planes of reflections (100), (002), (101), (102), (110), (103), and (112), respectively. The obtained data were strikingly similar to powder diffraction standard (JCPDS) card No. 036-1451 [31]. The XRD patterns of the synthesized nanoparticles employing the green procedure exhibit a comparable diffraction pattern without a significant peak shift. All of the peak positions characterized by diffraction patterns of ZnO-NPs are well matched to the diffraction pattern of the standard hexagonal crystal structure. The sharpness of the peaks in the spectra is the sign that nanoparticles were highly crystalline wherein the dissimilarity in particle sizes gave rise to different peak intensities. According to Scherrer's equation, the mean particle size of the synthesized ZnO-NPs using the diffraction peak of 36. 42° related with the (101) plane was 19 nm. The obtained pattern that appeared at 2*θ* positions was similar to those of the previously reported literature by Khatami et al. [23].

### 3.4. SEM Analysis of ZnO-NPs

SEM analysis was applied for the sample illustrations and considers the morphology of nanoparticles. A scanning electron micrograph depicted the shape and size of synthesized ZnO-NPs. This technique was also used to investigate the surface morphology and the formations of ZnO-NPs at various magnifications that are shown in Figure 4. The average diameter of ZnO-NPs was measured using ImageJ software (version 1.46), with the majority of the particles aggregated and polydispersed. However, a random spherical shape was confirmed from the given images, with an average particle diameter of 20-80 nm. This SEM result coincides with previously reported literature, which showed the formation of spherical-shaped nanoparticles [33]. Rajiv et al. synthesized ZnO-NPs in different sizes by using the *Parthenium hysterophorus L.* extract. They showed size-dependent biological properties of ZnO-NPs and stated that size change of particles can have an effect on properties of particles directly [23].

### 3.5. EDX Analysis of ZnO-NPs

Energy-dispersive X-ray analysis was carried out with a 20 keV accelerating voltage. The peaks in the EDX spectra for ZnO-NPs formed by employing 0.5 M ZnCl_2_ solution showed the synthesis of ZnO-NPs (Figure 5). The distribution of Zn and O in the EDX spectra was clearly visible, indicating the presence of ZnO in the analyzed particles. According to the quantitative results of the EDX spectrum of ZnO-NPs, the high-yield element Zn was observed in the L line, and these findings show a strong link to previously published research [34]. The elemental composition obtained from EDX analysis was zinc and oxygen at the plasmon resonance peak of 1 eV, 8.5 eV, and 0.5 eV, respectively. The appearance of a calcium peak suggests the unintentional accumulation of heavy metals inside the surface molecule of the plant extract, which is related to the composition of the soil [35, 36]. Parra and Haque reported similar findings, in which no other impurities such as C, N, or P were discovered. Therefore, ZnO nanoparticles were found to be nearly stoichiometric. This observation was in good agreement with the XRD results, which confirmed the phase purity of ZnO nanoparticles [37].

RETRACTED

### 3.6. Antidepressant Activity

#### 3.6.1. Effect of ZnO-NPs on Behavioral Analysis

The results of the antidepressant activity of the control group, depressive rats, plant extract of *S. procumbens*, precursor ZnCl_2Chem_, and ZnO-NPs are depicted in Figure 6. The immobility time was used to assess depressive behavior in rats as well as the efficacy of ZnO-NPs. Immobility is a sign of depression that manifests as a state of behavioral despair.  Figure 6(a) demonstrates the influence of ZnO-NP cure time of immobility in the forced swim test. According to the findings, ZnO-NPs significantly decrease the time of immobility (39.2%) compared to the control (40%). The immobility time of the ZnO-NP group was analogous to that of rats in the control group. In the tail suspension test, zinc oxide nanoparticle-treated rats had a significantly decreased immobility time (40%) in contrast to the control group (80%), as shown in Figure 6(b) and Table 1. The effects of tail suspension tests and forced swim tests indicate that ZnO-NPs have enhanced *in vivo* antidepressant activity [38, 39]. Alternatively, the increased activity may be an adaptive mechanism exerted by the brain to reduce the increase in acetylcholine levels. Several studies have recorded an increase in acetylcholine levels and linked this increase with the anxiety that was observed in depression [40].

#### 3.6.2. Effect of ZnO-NPs on BDNF Concentrations

The effect of ZnO-NPs on *in vivo* antidepressant activity was assessed by identifying the concentrations of BDNF in the brain and plasma. The findings in Table 2 revealed that reduction in the control group was observed in the BDNF concentration of the brain and plasma if opposed to other groups.  Figure 7(a) shows the result of treated ZnO-NPs that increased the plasma BDNF concentration (44%) compared to control (19.37%). The brain BDNF concentration of the ZnO-NP group (42.5%) was also higher than that of the control (18.52%) in Figure 7(b) and Table 2. It is important to realize that after ZnO-NP treatment, plasma and brain BDNF concentrations were nearly equivalent to the control group. From the results, it was confirmed that ZnO-NPs successfully improved BDNF concentrations that are also consistent to the results obtained from behavioral despair tests [41, 42]. Likewise, Khadrawy et al. used curcumin-coated iron oxide nanoparticles as antidepressive agents that are effective; most of them have intolerable side effects and delayed onset of therapeutic action [43].

RETRACTED

### 3.7. Cytotoxicity Results

The biocompatibility of zinc oxide nanoparticles with blood is more significant for its effective implementation. The dose applicability of ZnO-NPs at various concentrations (1, 3, 5, 7, 9, and 11 *μ*g) is shown in Table 3. For the positive control, the antidepressant fluoxetine was used, and DMSO was used for the negative control. The result of cytotoxicity exhibited that the dose (7 *μ*g) of ZnO-NPs demonstrated a significant antidepressant efficacy in rats. It is assumed that *S. procumbens* aqueous plant extract NPs are suggested to enhance bioavailability by increasing permeability and protecting it from the metabolism of the gut. ZnO-NPs are also known to improve the oral dosage absorption rate by gaining access to the lymphatic system via gut-associated lymphoid tissue and M-cells (which consists of lymphoidal follicles that form Peyer's patches) by enhancing chylomicron production and transport through triglyceride-rich lipoproteins [44]. However, higher doses (9 and 11 *μ*g) of ZnO-NP-treated groups showed a significant difference between the cell visibilities of other dose concentrations. In other words, the dose concentrations at 1, 3, and 5 *μ*g ZnO-NP-treated samples were not considerably different from that at 7 *μ*g. According to the data, a remarkably similar pharmacological effect was observed at doses 25 times lower than the dose at 7 *μ*g. Alternatively, the antidepressant activities of *S. procumbens* zinc oxide nanoparticle doses were gradually improved. Thus, the present NPs show good biocompatibility up to 11 *μ*g/mL (ZnO-NPs: 4.1%), and beyond this limit, the % cell visibility exceeded the permissible limit, as 5% cell visibility is permissible according to ASTM-E252408 for biomaterials [45].

RETRACTED

### 3.8. Proposed Mechanism for the Synthesis of ZnO-NPs

According to the reported literature, the phytochemicals present in *S. procumbens* are alkamides, phenolic groups, proteins, terpenoid groups, chlorogenic acid, 3,5-O-caffeoylquinic acid, and quercitrin [21, 22]. However, the exit mechanism of the metal nanoparticle by using plant extract is unknown due to the complex chemical composition of the plant extract. However, on the basis of the above observation, we can propose a general mechanism for the synthesis of ZnO-NPs as shown in Scheme 1. The reduction of Zn^2+^ to Zn^0^ is due to the existence of their functional biomolecules. The phenolic groups like chlorogenic acid, 3,5-O-caffeoylquinic acid, and quercitrin act as a reducing agent while proteins and alkamides and some other phytoconstituent present in the plant extract act as a capping agent for the ZnO-NP synthesis. The quercetin group present in adequate amount in *S. procumbens* plant extract acts as a better reducing agent. The –OH groups in quercetin may be responsible for releasing electrons during the bioreduction of Zn^2+^ to Zn^0^. The green synthesis of ZnO-NPs was catalyzed by the transition of electrons from the –OH groups of quercetin to reducible Zn^2+^ ions. The FT-IR analysis also supports this prediction that specifically showed that the presence of the –OH and –NH groups helps in the synthesis and stabilization of ZnO-NPs. During the reduction of the Zn ion, the enol form is converted into the keto form, and the charge-transfer-induced molecular changes in the polyphenolic groups are shown Scheme 1. The elimination of hydrogen atoms from the enol form allowed for the deduction of electrons that reduce Zn^2+^.

## 4. Conclusion

In the current investigation, the synthesis of ZnO-NPs was achieved by using an aqueous plant extract of *S. procumbens* that served as a reducing and stabilizing agent. The optical properties, crystalline nature, morphology, and elemental composition of ZnO-NPs were characterized by different techniques. The results showed that the prepared ZnO-NPs exhibit a significant antidepressant activity that was observed via the immobility time and BDNF concentration in the brain and plasma. Furthermore, the biocompatibility of ZnO-NPs as an antidepressant drug increases if the concentration increases. Furthermore, we suggest that future studies should also continue investigating alternative means of extending the effects of antidepressants or even replacing the nanoparticles that were used as antidepressants. It is also necessary to explore the proposed mechanisms of action that enhance prefrontal plasticity.

## Figures and Tables

**Figure 1:** UV-visible spectra of synthesized ZnO-NPs and plant extract of *S. procumbens*.

RETRACTED

**Figure 2:** (a) FT-IR spectra of plant extract *S. procumbens* and (b) synthesized ZnO-NPs.

**Figure 3:** XRD patterns of synthesized zinc oxide nanoparticles.

**Figure 4:** SEM image of synthesized ZnO-NPs.

**Figure 5:** EDX spectrum for ZnO nanoparticles.

**Figure 6:** Effects of ZnO-NPs on immobility time in the forced swim test (a) and the tail suspension test (b).

**Figure 7:** BDNF concentrations in plasma (a) and brain (b).

**Scheme 1:** Proposed mechanism for the synthesis of ZnO-NPs.

**Table 1:** Immobility time in (% reduction) FST and TST for depression.

Groups	% reduction for FST (w.r.t control)	% reduction for TST (w.r.t control)
Control	40	80
Depressive (dep.)	10	5.6
Dep.+ZnCl_2_	24	16
Dep.+extract	23.2	20.8
Dep.+ZnO-NPs	39.2	40.4

**Table 2:** BDNF concentrations (% reduction) in plasma and brain for depression.

Groups	% reduction for plasma (w.r.t control)	% reduction for brain (w.r.t control)
Control	19.37	18.52
Depressive (dep.)	87.25	86.2
Dep.+ZnCl_2_	71.25	70.3
Dep.+extract	70	69.2
Dep.+ZnO-NPs	44	42.5

**Table 3:** Cytotoxicity of synthesized zinc oxide nanoparticles.

S. no.	Sample (*μ*g/mL)	Cell visibility (%)
1	Fluoxetine	+ve control
2	DMSO	−ve control
3	1.0	1.51
4	3.0	2.6
5	5.0	3.0
6	7.0	4.1
7	9.0	5.7
8	11	8.4

## Data Availability

All the data supporting the results of our study is already incorporated in the main manuscript.

## References

[1] Mishra B., Patel B. B., Tiwari S. (2010). Colloidal nanocarriers: a review on formulation technology, types and applications toward targeted drug delivery. *Nanomedicine: Nanotechnology, Biology and Medicine*.

[2] Khan S. A., Shahid S., Lee C. S. (2020). Green synthesis of gold and silver nanoparticles using leaf extract of Clerodendrum inerme; characterization, antimicrobial, and antioxidant activities. *Biomolecules*.

[3] Bedi P., Kaur A. (2015). An overview on uses of zinc oxide nanoparticles. *World Journal of Pharmacy and Pharmaceutical Sciences*.

[4] Muhammad W., Ullah N., Haroon M., Abbasi B. H. (2019). Optical, morphological and biological analysis of zinc oxide nanoparticles (ZnO NPs) using Papaver somniferum L. *RSC Advances*.

[5] Sher M., Khan S. A., Shahid S. (2021). Synthesis of novel ternary hybrid g-C_3_N_4_@Ag-ZnO nanocomposite with Z-scheme enhanced solar light‐driven methylene blue degradation and antibacterial activities. *Journal of Environmental Chemical Engineering*.

[6] Tiloke C., Anand K., Gengan R. M., Chuturgoon A. A. (2018). Moringa oleifera and their phytonanoparticles: potential antiproliferative agents against cancer. *Biomedicine and Pharmacotherapy*.

RETRACTED

[7] Hanley C., Layne J., Punnoose A. (2008). Preferential killing of cancer cells and activated human T cells using ZnO nanoparticles. *Nanotechnology*.

[8] Reynolds I. S., Rising J. P., Coukell A. J., Paulson K. H., Redberg R. F. (2014). Assessing the safety and effectiveness of devices after US Food and Drug Administration approval: FDA-mandated postapproval studies. *JAMA International Medicine*.

[9] Fu P. P., Xia Q., Hwang H. M., Ray P. C., Yu H. (2014). Mechanisms of nanotoxicity: generation of reactive oxygen species. *Journal of Food and Drug Analysis*.

[10] Chen P., Wang H., He M., Chen B., Yang B., Hu B. (2019). Size-dependent cytotoxicity study of ZnO nanoparticles in HepG2 cells. *Ecotoxicology and Environmental Safety*.

[11] Amin F., Khattak B., Alotaibi A. (2021). Green synthesis of copper oxide nanoparticles using Aerva javanica leaf extract and their characterization and investigation of in vitro antimicrobial potential and cytotoxic activities. *Evidence-based Complementary and Alternative Medicine*.

[12] Nagaraju G., Nagabhushana H., Suresh D., Anupama C., Raghu G. K., Sharma S. C. (2017). *Vitis labruska* skin extract assisted green synthesis of ZnO super structures for multifunctional applications. *Cerâmica*.

[13] Singh A., Gautam P. K., Verma A. (2020). Green synthesis of metallic nanoparticles as effective alternatives to treat antibiotics resistant bacterial infections: a review. *Biotechnology. Reports*.

[14] Shanker K., Naradala J., Mohan G. K., Umar G. S., Pravallika P. L. A. (2017). A sub-acute oral toxicity analysis and comparative in vivo anti-diabetic activity of zinc oxide, cerium oxide, silver nanoparticles, and *Momordica charantia* in streptozotocin-induced diabetic Wistar rats. *RSC Advances*.

[15] Elumalai K., Velmurugan S. (2015). Green synthesis, characterization and antimicrobial activities of zinc oxide nanoparticles from the leaf extract of *Azadirachta indica* (L.). *Applied Surface Science*.

[16] Boima V., Tetteh J., Yorke E. (2020). Older adults with hypertension have increased risk of depression compared to their younger counterparts: evidence from the World Health Organization study of Global Ageing and Adult Health Wave 2 in Ghana. *Journal of Affective Disorder*.

[17] Seligman F., Nemeroff C. B. (2015). The interface of depression and cardiovascular disease: therapeutic implications. *Annals of the New York Academy of Sciences*.

[18] Ekambaram P., Sathali A. H., Priyanka K. (2012). Solid lipid nanoparticles. *Science Review and Chemical Communication*.

[19] Bal U., Touraev A. (2009). Microspore embryogenesis in selected medicinal and ornamental species of the Asteraceae. *Haploid Production in Higher Plants*.

RETRACTED

[20] Perez-Ochoa M. L., Chavez-Servia J. L., Vera-Guzman A. M., Aquino-Bolanos E. N., Carrillo-Rodriguez J. C. (2016). Medicinal plants used by indigenous communities of Oaxaca, Mexico, to treat gastrointestinal disorders. *Pharmacognosy Medicinal Plants*.

[21] Rios M. Y. (2012). Natural alkamides: pharmacology, chemistry and distribution. *Drug Discovery Research Pharmaceutical*.

[22] Wang L., Wang T., Guo Q. S., Huang Y., Xu H. K. (2013). Comparative study on four major active compounds of *Sanvitalia procumbens* and *Chrysanthemum morifolium* cv 'Hangju' and 'Gongju. *China Journal of Chinees Material and. Medicine*.

[23] Rajiv P., Rajeshwari S., Venkatesh R. (2013). Bio-fabrication of zinc oxide nanoparticles using leaf extract of *Parthenium hysterophorus L*. and its size-dependent antifungal activity against plant fungal pathogens. *Spectrochimica Acta Part A: Molecular and Biomolecular Spectroscopy*.

[24] Rana N., Khan M. M., Ansari F. A. (2020). Solid lipid nanoparticles-mediated enhanced antidepressant activity of duloxetine in lipopolysaccharide-induced depressive model. *Colloids and Surfaces. B, Biointerfaces*.

[25] Fitzgerald P. J., Hale P. J., Ghimire A., Watson B. O. (2020). The cholinesterase inhibitor donepezil has antidepressant-like properties in the mouse forced swim test. *Translational Psychiatry*.

[26] Can A., Dao D. T., Terrillion C. E., Piantadosi S. C., Bhat S., Gould T. D. (2011). The tail suspension test. *Journal of Visualized Experiments*.

[27] Najoom S., Fozia F., Ahmad I. (2021). Effective antiplasmodial and cytotoxic activities of synthesized zinc oxide nanoparticles using *Rhazya stricta* leaf extract. *Evidence-based Complementary and Alternative Medicine*.

[28] Aslam M., Fozia F., Gul A. (2021). Phyto-extract-mediated synthesis of silver nanoparticles using aqueous extract of *Sanvitalia procumbens*, and characterization, optimization and photocatalytic degradation of azo dyes orange G and direct blue-15. *Molecules*.

[29] Khan S. A., Shahid S., Shahid B., Fatima U., Abbasi S. A. (2020). Green synthesis of MnO nanoparticles using abutilon indicum leaf extract for biological, photocatalytic, and adsorption activities. *Biomolecules*.

[30] Ijaz F., Shahid S., Khan S. A., Ahmad W., Zaman S. (2017). Green synthesis of copper oxide nanoparticles using Abutilon indicum leaf extract: antimicrobial, antioxidant and photocatalytic dye degradation activitie. *Tropical Journal of Pharmaceutical Research*.

[31] Suresh D., Shobharani R. M., Nethravathi P. C., Kumar M. P., Nagabhushana H., Sharma S. C. (2015). Artocarpus gomezianus aided green synthesis of ZnO nanoparticles: luminescence, photocatalytic and antioxidant properties. *Acta Part A Molecules of Biomolecular Spectroscopy*.

RETRACTED

[32] Khatami M., Alijani H. Q., Heli H., Sharifi I. (2018). Rectangular shaped zinc oxide nanoparticles: green synthesis by Stevia and its biomedical efficiency. *Ceramics International*.

[33] Satdeve N. S., Ugwekar R. P., Bhanvase B. A. (2019). Ultrasound assisted preparation and characterization of Ag supported on ZnO nanoparticles for visible light degradation of methylene blue dye. *Journal of Molecular Liquids*.

[34] Aminuzzaman M., Ying L. P., Goh W. S., Watanabe A. (2018). Green synthesis of zinc oxide nanoparticles using aqueous extract of *Garcinia mangostana* fruit pericarp and their photocatalytic activity. *Bulletin of Materials Science*.

[35] Singh R., Gautam N., Mishra A., Gupta R. (2011). Heavy metals and living systems: an overview. *Indian Journal of Pharmacology*.

[36] Keshtkar M., Dobaradaran S., Soleimani F., Karbasdehi V. N. (2016). Data on heavy metals and selected anions in the Persian popular herbal distillates. *Data in Brief*.

[37] Parra M. R., Haque F. Z. (2014). Aqueous chemical route synthesis and the effect of calcination temperature on the structural and optical properties of ZnO nanoparticles. *Journal of Materials Research and Technology*.

[38] Yankelevich Y. R., Franko M., Huly A., Doron R. (2015). The forced swim test as a model of depressive-like behavior. *Journal of Visualized Experiments*.

[39] Stukalin Y., Lan A., Einat H. (2020). Revisiting the validity of the mouse tail suspension test: systematic review and meta-analysis of the effects of prototypic antidepressants. *Neuroscience and Biobehavioral Reviews*.

[40] Mineur Y. S., Obayemi A., Wigestrand M. B. (2013). Cholinergic signaling in the hippocampus regulates social stress resilience and anxiety- and depression-like behavior. *Proceedings of the National Academy of Sciences*.

[41] Mannari C., Origlia N., Scatena A. (2008). BDNF level in the rat prefrontal cortex increases following chronic but not acute treatment with duloxetine, a dual acting inhibitor of noradrenaline and serotonin re-uptake. *Cellular and Molecular Neurobiology*.

[42] Hutten N. R., Mason N. L., Dolder P. C. (2021). Low doses of LSD acutely increase BDNF blood plasma levels in healthy volunteers. *ACS Pharmacology and Translational Science*.

[43] Khadrawy Y. A., Hosny E. N., Magdy M., Mohammed H. S. (2021). Antidepressant effects of curcumin-coated iron oxide nanoparticles in a rat model of depression. *European Journal of Pharmacology*.

[44] Shewale P. B., Patil R. A., Hiray Y. A. (2012). Antidepressant-like activity of anthocyanidins from Hibiscus rosa-sinensis flowers in tail suspension test and forced swim test. *Indian Journal of Pharmacology*.

RETRACTED

[45] Zuraidah M. A., John B. A., Kamaruzzaman Y. (2017). Cytotoxicity on MCF7 cell lines exposed to an extract of the jacalin from jackfruit seed. *Science Heritage Journal*.

